# Roles of microRNAs in inflammatory bowel disease

**DOI:** 10.7150/ijbs.59904

**Published:** 2021-05-17

**Authors:** HyunTaek Jung, Jae Seok Kim, Keum Hwa Lee, Kalthoum Tizaoui, Salvatore Terrazzino, Sarah Cargnin, Lee Smith, Ai Koyanagi, Louis Jacob, Han Li, Sung Hwi Hong, Dong Keon Yon, Seung Won Lee, Min Seo Kim, Paul Wasuwanich, Wikrom Karnsakul, Jae Il Shin, Andreas Kronbichler

**Affiliations:** 1 Yonsei University College of Medicine, Seoul, Republic of Korea.; 2 Department of Nephrology, Yonsei University Wonju College of Medicine, Wonju, Republic of Korea.; 3 Department of Pediatrics, Yonsei University College of Medicine, Seoul, Republic of Korea.; 4 Laboratory Microorganisms and Active Biomolecules, Sciences Faculty of Tunis, University Tunis El Manar, Tunis, Tunisia.; 5 Department of Pharmaceutical Sciences and Interdepartmental Research Center of Pharmacogenetics and Pharmacogenomics (CRIFF), University of Piemonte Orientale, Novara, Italy.; 6 The Cambridge Centre for Sport and Exercise Science, Anglia Ruskin University, Cambridge, CB1 1PT, UK.; 7 Research and Development Unit, Parc Sanitari Sant Joan de Déu, CIBERSAM, 08830 Barcelona, Spain.; 8 ICREA, Pg. Lluis Companys 23, 08010 Barcelona, Spain.; 9 Faculty of Medicine, University of Versailles Saint-Quentin-en-Yvelines, 78000 Versailles, France.; 10 University of Florida College of Medicine, Gainesville, FL 32610, USA.; 11 Department of Pediatrics, Seoul National University Children's Hospital, Seoul National University College of Medicine, Seoul, Republic of Korea.; 12 Department of Data Science, Sejong University College of Software Convergence, Seoul, Republic of Korea.; 13 Korea University, College of Medicine, Seoul, Republic of Korea.; 14 Division of Pediatric Gastroenterology, Hepatology, and Nutrition, Department of Pediatrics, Johns Hopkins University School of Medicine, Baltimore, USA.; 15 Department of Internal Medicine IV (Nephrology and Hypertension), Medical University Innsbruck, Innsbruck, Austria.

**Keywords:** inflammatory bowel diseases, Crohn's disease, ulcerative colitis, microRNAs

## Abstract

Inflammatory bowel disease (IBD) is a chronic inflammatory disease of the gastrointestinal tract that mainly affects young people. IBD is associated with various gastrointestinal symptoms, and thus, affects the quality of life of patients. Currently, the pathogenesis of IBD is poorly understood. Although intestinal bacteria and host immune response are thought to be major factors in its pathogenesis, a sufficient explanation of their role in its pathophysiologic mechanism has not been presented. MicroRNAs (miRNAs), which are small RNA molecules that regulate gene expression, have gained attention as they are known to participate in the molecular interactions of IBD. Recent studies have confirmed the important role of miRNAs in targeting certain molecules in signaling pathways that regulate the homeostasis of the intestinal barrier, inflammatory reactions, and autophagy of the intestinal epithelium. Several studies have identified the specific miRNAs associated with IBD from colon tissues or serum samples of IBD patients and have attempted to use them as useful diagnostic biomarkers. Furthermore, some studies have attempted to treat IBD through intracolonic administration of specific miRNAs in the form of nanoparticle. This review summarizes the latest findings on the role of miRNAs in the pathogenesis, diagnosis, and treatment of IBD.

## Introduction

Inflammatory bowel disease (IBD) is a complex and multifactorial condition characterized by chronic gastrointestinal tract inflammation. There are two main forms of IBD: Crohn's disease (CD) and ulcerative colitis (UC). CD is manifested as patchy transmural inflammatory patterns that affect all layers of the intestinal wall in any portion of the gastrointestinal tract, whereas UC is limited to the innermost layers of the mucosa in the large intestine. CD and UC mainly affect young people, causing bloody diarrhea, abdominal pain, malabsorption, fatigue, and impaired quality of life 1. Long-lasting inflammation also increases the risk of colorectal cancer in patients with IBD, which has a mortality rate of 10-15% 2.

Rapid modernization and urbanization seem to be related to the increasing incidence of IBD, which affects approximately 0.5% of the general population in developed nations 3, 4; however, the exact pathogenesis of IBD remains poorly understood. Based on speculations, IBD is presumed to be the result of complex interactions among genetic, microbial, and environmental factors 1. Genome-wide association studies (GWASs) have identified the genetic susceptibility loci for IBD, and more than 240 of these loci have been reported 5-8. Substantial differences have been found between different ethnic groups 9, 10. Moreover, the existence of IBD susceptibility mutations is not sufficient to explain the entire disruption of intestinal homeostasis; this is because twin studies revealed low concordance between genetic variations and clinical presentation of the disease 11. The role of the microbiome and lifestyle factors in the pathogenesis of IBD is unquestionable; however, these conditions only cause disease in genetically susceptible individuals 12.

Recent molecular research has shown that microRNAs (miRNAs or miR-) play important roles in the pathophysiology of IBD 13. miRNAs are evolutionarily conserved, endogenous, single-stranded, non-coding RNAs that bind to the 3' untranslated region (UTR), 5' UTR, or partially translated region of a target mRNA, inhibiting mRNA translation and blocking its expression 14. miRNAs are major regulators of cell function and homeostasis, and their abnormal activity has been demonstrated in various diseases, including IBD. Thus, novel treatment options could be developed to alter imbalances in miRNA expression by targeting certain molecular pathways 15. In this study, we evaluated the role of miRNAs in IBD by examining published results of studies conducted in the past 2-3 years and suggest the clinical potential of miRNAs as biomarkers and/or new therapeutic strategies for IBD.

## Biosynthesis of microRNA

miRNAs are small, 18-21 nucleotide-long, evolutionarily conserved RNA molecules involved in the regulation of gene expression. The primary nuclear transcripts of miRNAs, or pri-miRNAs, are typically a few thousand nucleotides long and are located in introns, exons, or intergenic regions of the human genome. Pri-miRNAs are processed into 70 nucleotide-long, stem-loop structured pre-miRNAs by the RNAse-3-type enzyme Drosha. Pre-miRNAs are then translocated to the cytosol from the nucleus and cleaved by the endoribonuclease Dicer. The remaining miRNA duplex binds with Argonaute to form an RNA-induced silencing complex (RISC). The guidance strand directs the RISC to the complementary region in the 3'-UTR of the target mRNA, and the RISC makes post-transcriptional modifications. When an exact match is found, the target mRNA is degraded; however, when an incomplete match occurs, translation is destabilized 14. **Figure 1** briefly summarizes the biosynthesis of miRNAs and their mechanisms of action.

The seed region responsible for identifying target mRNAs is a 6 nucleotide-long sequence from the 2nd to the 7th nucleotide of the miRNA. Based on similar seed sequences, miRNAs are classified into miRNA families. Members of a given miRNA family share almost the same pool of mRNAs as their target as they possess the same seed region. Numerous miRNAs form clusters in the genome and are transcribed as one common pri-miRNA; therefore, their transcription is regulated simultaneously. Notably, the role of miRNAs is redundant; multiple different miRNAs can control a single mRNA, and a given miRNA can inhibit numerous mRNAs. miRNA regulation does not act as a switch; rather, it functions as a synchronized tuner of gene expression 16.

## Brief description of the pathophysiology of IBD

Commensal bacteria are essential components in the maintenance of intestinal homeostasis. They provide essential nutrients, assist in energy metabolism, and suppress the growth of pathogenic bacteria by competitive inhibition in the intestine 17. Nevertheless, they can cause opportunistic infections and are under the surveillance of host immunity. Consequently, the human immune system has adapted to maintain a commensal relationship by establishing a balance between immune suppression and activation. The intestine is continuously exposed to large amounts of toxins and antigenic proteins from ingested foods. Therefore, a high level of immune tolerance is essential for intestinal homeostasis 18. However, well-controlled immune responses can be aberrantly activated by altered states of intestinal bacteria or the intestinal barrier, which are two important factors that maintain immune tolerance. From our perspective, a disruption in physiological balance can result in the development of IBD (**Figure 2**).

Many immune cells, such as neutrophils, dendritic cells, macrophages, and lymphoid cells, reside in the intestinal epithelium and the underlying lamina propria. These cells are regulated by immune tolerance mechanisms. When macrophages phagocytose the antigen from commensal bacteria, interleukin (IL)-10 is secreted from macrophages 19, resulting in the promotion of the response of a cluster of differentiation 4^+^ (CD4^+^) Treg cells to suppress inflammatory T cell reactions. CD4^+^ Treg cells produce IL-10 and transforming growth factor β1 (TGF-β1) to change the subtype of macrophages into an anti-inflammatory phenotype and to facilitate peripheral development of Treg cells 20. Serum amyloid A is an important acute reactant protein produced in the intestine and liver. A previous study demonstrated that serum amyloid A had a higher increase in the presence of intestinal microbiota than in the germ-free state. Serum amyloid A enhances the recruitment of neutrophils to the intestine and increases pro-inflammatory gene expression in neutrophils, but decreases bactericidal capability and inflammatory tones 21, 22. These contradictory responses would not damage the intestinal microbiota during the prevention of opportunistic infections by commensal bacteria. CD4^+^ T cells secrete IL-21 and TGF-β1 to stimulate immunoglobulin (Ig) class switching in B cells. The secreted IgAs bind to commensal bacteria in the intestinal lumen, which prevents bacteria from invading the intestinal epithelium, and suppress the inflammatory reaction of the intestinal barrier against commensal bacteria 23. Retinoic acid, a metabolite of vitamin A, is an important nutritional factor that is closely related to the immune response. Retinoic acid plays an important role in maintaining intestinal homeostasis, specifically inducing intestinal immune tolerance through the actions of CD103^+^ dendritic cells and innate lymphoid cells (ILCs)3 24. However, based on a recent study, commensal bacteria reduced retinoic acid and IL-22 by inhibiting retinol dehydrogenase 7 (Rdh7) in intestinal epithelial cells. Consequently, the anti-microbial reaction was downregulated, and a symbiotic state could be maintained 25. Such findings indicate that retinoic acid has both tolerogenic capacity and antimicrobial activity. Thus, intestinal immune tolerance does not simply mean a decrease in intestinal immunity, but rather a balanced state in which anti-inflammatory and anti-microbial activities coexist. The aryl hydrocarbon receptor (AhR) is a transcription factor that induces anti-inflammatory reactions at the gene level. Previous studies have indicated that AhR reduces intestinal inflammation through anti-inflammatory mediators, such as IL-10 and IL-22. Several AhR ligands exist in the intestine, the majority of which are metabolites of commensal bacteria. Therefore, intestinal microbiota contributes to AhR-induced immunomodulation 26, 27. Taken together, host immunity has dual effects on the intestinal microbiota to maintain intestinal homeostasis. The intestinal immune system should maintain an appropriate balance between inflammatory and anti-inflammatory responses. Dysbiosis, which is an imbalance in microbes in the intestine, disrupts intestinal homeostasis and should thus be considered as a major cause of IBD 28.

The intestinal epithelium is one of the key components that sustain homeostasis of the intestine. The membranous barrier separates intestinal germs from the submucosal lymphoid tissue to prevent inflammatory responses and integrates molecular signals from dietary metabolites, commensal bacteria, and pathogens to regulate immune reactions 29. Resident lymphoid cells, such as NK T cells, γδ T cells, ILCs, intraepithelial lymphocytes, and CD8^+^ mucosal-associated invariant T cells produce IL-6, IL-17, and IL-22 to activate the signal transducer and activator of transcription (STAT) 3 pathway in response to disruption of the intestinal barrier. The STAT3 pathway promotes the recovery of barrier function and increases mucus secretion and epithelial repair 30. Macrophages secrete type I interferon (IFN) and activate STAT1 and STAT2 pathways to prevent epithelial apoptosis, promote epithelial differentiation, and maintain the integrity of the intercellular barrier 31. CD4^+^ T cells produce IL-17 and IL-22 in response to IL-23 and serum amyloid A, which results in the activation of the STAT3 pathway in the epithelium 32. These interactions enhance the intestinal barrier against pathogenic luminal bacteria.

When the mucus barrier is broken, permeability through the epithelium increases. These situations are mostly due to the dysfunction of the mucosal barrier itself, or inflammatory damage. Mucous membrane disorder, tight junction disorder, increased intestinal permeability, and increased binding of bacteria to epithelial cells can induce intestinal inflammation. Penetration of intestinal bacteria, including intestinal microbiota, into the lamina propria leads to recognition by phagocytes and the production of inflammatory cytokines by macrophages. Macrophages secrete IL-1β to promote the differentiation of CD4^+^ T cells into T helper 17 (Th17) cells and the production of IFN-γ 33, 34. Damaged epithelium releases IL-18, which disrupts goblet cell maturation and impairs its function, leading to further damage of the membranous barrier 35. Macrophages enhance the survival of pro-inflammatory T cells and stimulate epithelial apoptosis through the tumor necrosis factor-α (TNF‐α) signaling pathway 36, 37. IL-6 from macrophages and granulocyte-macrophage colony-stimulating factor (GM-CSF) from ILCs recruit polymorphonuclear leukocytes, which secrete pro-inflammatory cytokines for pathogenic T cell responses 38-40. Repeated cycles of dysregulated immune responses result in chronic intestinal injury and fibrotic remodeling in patients with IBD 41.

IBD is a multifactorial disease. Although dysbiosis of commensal bacteria and breakdown of the intestinal barrier are considered as major pathological mechanisms in the development of IBD, other important factors such as genetic aberrations also contribute to its development. In this regard, miRNAs are an emerging risk factor for IBD. miRNAs are involved in the maintenance of intestinal barrier integrity, as well as a large number of intracellular signaling pathways involved in inflammatory or anti-inflammatory actions 42.

## Role of miRNAs in the pathophysiology of IBD

miRNAs have been reported to be associated with several pathophysiological factors of IBD. miRNAs affect the intestinal barrier and inflammatory reactions through various pathological mechanisms. The pathogenic roles of miRNAs in IBD are summarized in **Table 1**.

### miRNAs and the intestinal barrier in IBD

Disrupted intestinal membranes are one of the most significant factors in the pathogenesis of IBD. TNF-α is known to be a major pro-inflammatory cytokine in the pathogenesis of IBD. Therefore, several *in vitro* experiments have been conducted using intestinal epithelial cells to induce injury by TNF-α 43. miR-191a and miR-212 are known to damage intestinal barriers. In fact, *in vitro* studies have shown that their mimics downregulate the expression of zonula occludens (ZO)-1, one of the major components of the tight junction between the intestinal epithelium 44, 45. By measuring the binding of miR-675 in colon cells *in vitro*, Zou et al. found that miR-675 destabilized the mRNA of ZO-1 and cadherin E, causing reduced expression of key molecules for intercellular tight junctions 46. Aquaporin 3 is another important protein in the intestinal membrane. The overexpression of miR-874 *in vitro* induced by pre-miR-874 transfection in intestinal epithelial cells was demonstrated to decrease the expression of aquaporin 3 47. Epidermal growth factor receptor (EGFR) was identified as the target gene of miR-122a. The overexpression of miR-122a was found to increase zonulin expression and intestinal permeability 48. Further, the overexpression of miR-21 *in vitro* was found to cause an increase in intestinal barrier defects and was suggested to target the phosphatase and tensin homolog (PTEN)/PI3K (phosphoinositide 3-kinase)/Akt signaling pathway to enhance the paracellular permeability of the intestinal epithelium 49. As the miR-21 mimic suppressed the level of PTEN and increased the level of phospho-Akt (p-Akt) *in vitro*, Zhang et al. reported the impairing of intestinal permeability through the PTEN/PI3K/Akt pathway as a potential mechanism 49.

Some miRNAs have been reported to strengthen the intestinal barrier. Transfection of the miR-200b precursor in TNF-α-treated intestinal epithelium *in vitro* inhibited the damage to trans-epithelial electrical resistance and intercellular tight junctions. Further, c-Jun and myosin light chain kinase (MLCK) were demonstrated to be the targets of miR-200b 50. Haines et al. revealed that silencing the expression of protein tyrosine kinase 6 (PTK6) with miR-93 in the intestinal epithelium increased the resistance to TNF-α-induced injury 51.

### miRNAs and immune response in IBD

miRNAs are known to contribute to the immunological reactions that lead to IBD. Shi et al. compared miR-21 knockout mice to wild-type mice after the induction of intestinal damage by dextran sulfate sodium (DSS); miR-21 knockout mice demonstrated reduced weight loss, intestinal inflammation (confirmed by histopathology), serum leukocyte levels, and TNF-α and macrophage inflammatory protein 2 (MIP2) levels in colon culture supernatants compared to wild-type mice 52. miR-124 was reported to target the 3'-UTR of AhR to suppress its expression in Caco-2 cells and HT-29 cells *in vitro* 53. Intracolonic administration of miR-124 inhibitors and precursors to 2,4,6-trinitrobenzen acid (TNBS)-induced colitis mice was found to alleviate and aggravate intestinal inflammation, respectively 53.

Some miRNAs have been reported to suppress intestinal inflammation. Nucleotide-binding oligomerization domain-containing protein 2 (NOD2) is one of the genes clearly associated with CD 54. In fact, Pierdomenico et al. reported its relationship with miR-320 55. HT29 cells transfected with exogenous miR-320 displayed a downregulated expression of NOD2, while miR-320 inhibitor increased NOD2 expression as well as its downstream signaling pathway, leading to nuclear factor κB (NF-κB) and inflammatory cytokines 55. Wu et al. used human monocyte-derived dendritic cells and CD4^+^ T cells isolated from the peripheral blood of IBD patients treated with the miR-10a precursor. The transfection caused decreased expression of IL-12/23p40 (p40 subunit of IL-12 and IL-23) in dendritic cells and suppression of IFN-γ, TNF-α, and IL-17A in CD4^+^ T cells, suggesting inhibited differentiation into Th1 and Th17 cells 56. C-X-C motif chemokine ligand 12β (CXCL12β) is an important mediator of leukocyte migration. Huang et al. used TNBS-induced colitis mice, IL-10 knockout colitis mice, and colon biopsy samples of CD patients to identify an inverse relationship between miR-141 expression and CXCL12β levels 57. Intracolonic administration of miR-141 precursors and inhibitors to both TNBS-colitis mice and IL-10 knockout mice alleviated and aggravated colitis, respectively 57.

### miRNAs and autophagy in IBD

Autophagy is a cellular response that degrades and recycles internal structures, such as organelles and macromolecules. Therefore, its purpose is to maintain cell homeostasis and regulate inflammatory responses 58. Defects in autophagy can cause epithelial dysfunction and immune disruption, which play important roles in the pathogenesis of IBD 59. Recent studies suggest that miRNAs target autophagy-susceptibility genes to regulate intestinal autophagy and control intestinal inflammation in IBD 60. *ATG16L1* is an autophagy-related gene that forms autophagosomes during autophagy 61. miR-346 was reported to downregulate the expression of the vitamin D receptor, glycogen synthase kinase 3 beta (GSK3B), to increase the level of *ATG16L1* in colon biopsy samples of IBD patients 62. miR-665 represses X-box binding protein 1 (XBP1) and ORMDL sphingolipid biosynthesis regulator 3 (ORMDL3), which also stimulates autophagy 63.

Many miRNAs are known to inhibit autophagy. miR-20a downregulates Beclin 1 (BECN1), *ATG16L1*, and sequestosome 1 (SQSTM1), which collectively slows down autophagy 64. miR-30C 65, miR-93, miR-106B 66, 67, and miR-142-3p 68 also target the expression of *ATG16L1* to prevent autophagy. miR-122 69, miR-192 70, and miR-320 55 were found to decrease the activity of NOD2 to block autophagy. miR-130a increases the level of phosphorylated mammalian target of rapamycin (p-mTOR) 71, while miR-132, miR-223, miR-146b, and miR-155 reduce Forkhead box class O3 (FOXO3 or FOXO3a) to inhibit autophagy 72-76. miR-196 blocks the accumulation of the lipid-modified form of microtubule-associated protein 1A/1B-light chain 3 (LC3-II) to prevent autophagy 77.

## Role of miRNAs in IBD diagnosis

Diagnosis and evaluation of IBD have always been challenging. IBD is diagnosed based on clinical manifestations and endoscopy with histopathological examination 78; however, various clinical manifestations make diagnosis difficult, and endoscopy with histopathology requires the expertise of clinicians 79. As miRNAs are known to be associated with the pathogenesis of IBD, several studies have suggested that miRNAs are non-invasive and inexpensive biomarkers. A list of possible candidates is provided in **Table 2**.

### miRNA signature from the colon tissues of IBD patients

Some studies found abnormal elevation of miRNA levels in the mucosal tissues of UC patients compared to those of healthy controls. In fact, Wu et al. found that miR-16, miR-21, miR-23a, miR-24, miR-29a, miR-126, miR-195, and let-7f were upregulated in active UC patients compared to healthy controls 80. By comparing the colonic mucosa of UC patients and healthy controls, Fasseu et al. showed that miR-7, miR-26a, miR-29a, miR-29b, miR-31, miR-126* (the complement of miR-126), miR-127-3p, miR-135b, and miR-324-3p were increased in the inflamed mucosa of UC patients 81. Takagi et al. found increased levels of miR-21, miR-155, miR-923, let-7a, let-7c, let-7d, and let-7g in colon biopsy specimens of active UC patients compared to healthy controls 82. miR-126 83 and miR-150 84 were elevated in the colonic mucosa of patients with active UC compared to controls. Frozen biopsy samples of distal colectomy from UC patients were found to have significant increases in miR-31, miR-146a, miR-206, and miR-424 levels 85. Coskun et al. identified increases in miR-20b, miR-26b, miR-98, miR-99a, and miR-203 levels in colon biopsy samples of active UC patients compared to healthy controls, inactive UC patients, and CD patients 86.

Decreased levels of miR-188-5p, miR-215, miR-320a, and miR-346 were observed in the inflamed mucosa of UC patients compared to controls 81. miR-141 was found to be downregulated in the colonic mucosa of patients with active UC compared to healthy controls 87. miR-192, miR-375, and miR-422b were downregulated in colon biopsy samples from patients with active UC 80.

The mucosal tissue samples of patients with active CD had aberrant expression of miRNAs compared to controls. Fasseu et al. reported that miR-9, miR-21, miR-22, miR-26a, miR-29b, miR-29c, miR-30b, miR-31, miR-34c-5p, miR-106a, miR-126*, miR-127-3p, miR-130a, miR-133b, miR-146a, miR-146b-5p, miR-150, miR-155, miR-181c, miR-196a, miR-324-3p, and miR-375 were elevated in the inflamed mucosa of CD patients relative to levels in healthy controls 81. Further, Lin et al. showed that miR-31, miR-146a, miR-206, and miR-424 were increased in frozen biopsy samples of CD patients compared to controls, similar to that found in UC patients 85. miR-106b 66 and miR-196 77 were upregulated in the intestinal epithelium of patients with active CD compared to controls. Schaefer et al. found an increase in miR-31, miR-101, and miR-146a levels in colon biopsy samples from CD patients compared to healthy controls 88. Further, miR-7 and miR-375 levels were decreased in the actively inflamed colonic mucosa of CD patients 88, 89.

Among the miRNAs included in the differential analysis of IBD colon tissues, miR-21, miR-31, and miR-141 are suggested to be valuable targets for the diagnosis of IBD. miR-21 is known to be an important factor in the pathogenesis of IBD as it modulates T-cell responses 90 and disrupts intercellular tight junctions in the intestinal epithelium 91. miR-21 was found to be elevated in the mucosal tissue of both UC and CD 92, 93, and the knockout of miR-21 in a mouse model of DSS-induced colitis inhibited the inflammatory response and increased survival rate, indicating the importance of miR-21 in IBD 52. miR-31 was upregulated in the colon tissues of both UC and CD patients 88; this miRNA is known to target IL-25 to stimulate the Th1/Th17-mediated pro-inflammatory molecular pathway in mouse colitis models 94. miR-31 has also been suggested to be capable of distinguishing IBD from microscopic colitis, as its expression is elevated in IBD compared to microscopic colitis 95. miR-141 inhibits CXCL5 and CXCL12β, and its downregulation in IBD is expected to stimulate leukocyte recruitment and the consequent inflammatory response. A decrease in miR-141 was observed in the colon tissues of patients with UC 87.

Furthermore, useful findings have been obtained from the analysis of colon samples from patients with IBD. After acquiring rectal biopsy samples of UC and CD patients, Zham et al. found that miR-24 was increased in UC samples compared to CD samples, with a sensitivity of 83.3% and specificity of 85.7% as a diagnostic biomarker 96. Jeremy et al. used matched colon biopsies from UC and CD patients to compare endoscopically involved regions with endoscopically uninvolved regions of each patient. miR-21, miR-31, miR-101, miR-142-3p, miR-142-5p, miR-155, miR-223, miR-375, and miR-494 levels were elevated in active CD lesions compared to inactive regions; miR-21, miR-101, miR-142-5p, miR-146a, miR-155, and miR-223 levels were higher in active UC lesions than in inactive regions 88. Guo et al. compared inflamed and non-inflamed mucosal samples of the terminal ileum of active CD patients and found that miR-124-3p and miR-192-5p levels were decreased, while miR-361-3p was upregulated in the inflamed mucosa of CD patients 97.

### miRNA signature from the peripheral blood of IBD patients

As the acquisition of colon tissues requires a relatively invasive procedure compared to blood sampling, some studies have attempted to identify miRNA signatures from the peripheral blood of patients with active IBD. Paraskevi et al. reported increased levels of miR-16, miR-23a, miR-29a, miR-106a, miR-107, miR-126, miR-191, miR-199a-5p, miR-200c, miR-362-3p, and miR-532-3p in the blood of CD patients compared to healthy controls, and elevated levels of miR-16, miR-21, miR-28-5p, miR-151-5p, miR-155, and miR-199a-5p in the blood of UC patients compared to controls 98. Wu et al. found increased levels of miR-199a-5p, miR-340*, miR-362-3p, miR-532-3p, and miRplus-E1271, and decreased levels of miR-149* and miRplus-F1065 in the blood of patients with active CD compared to controls 99. The levels of miR-28-5p, miR-103-2*, miR-151-5p, miR-199a-5p, miR-340*, miR-362-3p, miR-532-3p, and miRplus-E1271 were increased, while that of miR-505* was decreased in the peripheral blood samples of active UC patients compared to healthy controls 99. By measuring miRNAs from the platelet fraction, Duttagupta et al. found increased levels of miR-188-5p, miR-378, miR-422a, miR-500, miR-501-5p, miR-769-5p, and miR-874 in blood samples from UC patients compared to controls 100. Schaefer et al. collected peripheral blood from UC and CD patients with normal controls and reported elevated levels of miR-19a, miR-101, miR-142-5p, miR-223, miR-375, and miR-494, and reduced levels of miR-21, miR-31, and miR-146a in the blood samples of UC patients compared to healthy controls; the levels of miR-101 and miR-375 were increased, while those of miR-21, miR-31, miR-146a, and miR-155 were decreased in the whole blood of CD patients compared to controls 88. Zahm et al. reported elevated levels of miR-16, miR-20a, miR-21, miR-30e, miR-93, miR-106a, miR-140, miR-192, miR-195, and miR-484 in serum samples from pediatric CD patients compared to normal controls 101.

Viennois et al. found that the levels of miR-29b-3p, miR-122-5p, miR-146a-3p, miR-150-5p, miR-192-5p, miR-194-5p, and miR-375-3p were elevated in the serum of IL10 (-/-) mice, which distinguished peripheral blood samples from UC patients and healthy controls with 83.3% sensitivity 102. Wu et al. reported that the serum levels of eight miRNAs (miR-28, miR-103-2*, miR-149*, miR-151, miR-340*, miR-505*, miR-532, and miR-plus-E1153) could be used to distinguish UC from CD 99. Jensen et al. used reverse-transcription polymerase chain reaction (RT-PCR) to measure the miRNA levels in serum samples of CD patients and healthy controls. Thereafter, they proposed that a decrease in serum miR-16b could be used to diagnose CD, which yielded an area under the curve of 65% 103. Zham et al. measured 11 miRNAs (miR-16, miR-20a, miR-21, miR-30e, miR-93, miR-106a, miR-140, miR-192, miR-195, miR-484, and let7b) in serum samples from CD patients and healthy controls and reported that their elevation served as a diagnostic marker for CD with a sensitivity of 70%-83% and specificity of 75%-101%. By performing miRNA microarray analysis of the saliva from UC patients, CD patients, and healthy controls, Schaefer et al. found increases in the levels of miR-21, miR-31, and miR-142-3p and a decrease in miR-142-5p levels in UC patients, while saliva samples from CD patients showed elevated miR-26a and miR-101 levels compared to controls 88.

Gallo et al. suggested that miRNAs in human saliva and serum samples mainly exist in the form of exosomes (encapsulated microvesicles) 104. Vickers et al. presented evidence that miRNAs are transported by high-density lipoprotein (HDL) to recipient cells 105. Exosomes and HDL can protect miRNAs from ribonucleases in the blood, which makes it easier to measure miRNA levels in serum samples.

## Role of miRNAs in the treatment of IBD

As *in vitro* studies have confirmed the importance of miRNAs in the pathophysiology of IBD, some researchers have attempted to administered miRNAs *in vivo* to mice with experimental colitis. Intracolonic administration of miRNA mimic molecules and antagonists led to the overexpression and inhibition of miRNA expression, respectively 106.

### Nanoparticle-mediated approach

Tian et al. found that the delivery of the miR-31 mimic into the colon of DSS-colitis mice alleviated the inflammatory response. miR-31 was bound to encapsulating microspheres and administered via enema, resulting in a slower loss of body weight and colon length, as well as increased epithelial proliferation and reduced inflammation, as confirmed by colon biopsy 107. Neudecker et al. also reported the attenuation of occult bleeding, weight loss, and edema in DSS-colitis mice after intracolonic administration of synthetic murine miR-223 mimetic in nanoparticle lipid emulsion 108. The intracolonic administration of miR-141 precursors in mice with TNBS-induced colitis resulted in a decrease in CXCL12β expression and leukocyte infiltration in the intestine 57. miR-146b was also found to alleviate intestinal inflammation when administered into the peritoneum of DSS-induced colitis mice with expression vectors 74. By using a mouse model of TNBS-induced colitis, Cheng et al. demonstrated that the intracolonic administration of pre-miR-19b can suppress the inflammatory process, with *in vitro* results suggesting that miR-19b inhibits suppressor of cytokine signaling 3 (SOCS3) to reduce inflammation of the intestinal epithelium in IBD 109. miR-200b bound to microvesicles was administered to intestinal epithelial cells *in vitro* and the colon of TNBS-colitis mice *in vivo*; this administration resulted in the attenuation of intestinal fibrosis with suppression of TGF-β1 mediated epithelium-to-mesenchyme transition 110.

Other routes of administration have been attempted to deliver miRNA mimic molecules to mice with colitis. Zhang et al. purified nanoparticles from edible ginger and found that their oral administration by colitis mice reduced the severity of colitis and promoted wound healing. The nanoparticles contained around 125 miRNAs. Further, the colon samples of mice administered the nanoparticles had a decrease in pro-inflammatory cytokines (TNF-α, IL-6, and IL-1β), increase in anti-inflammatory cytokines (IL-10 and IL-22), and increase in the proliferation of the epithelium based on the biopsy 111. Fukata et al. attempted to intravenously administer miR-29a-3p and miR-29b-3p bound to supercarbonate apatite. These researchers reported a decrease in the inflammatory response in DSS-colitis mice and revealed that the subcutaneous injection of miR-29b bound to supercarbonate apatite inhibited the immune response by targeting CD11c^+^ dendritic cells in a DSS-colitis model 112.

## Conclusion

IBD is a multifactorial disease associated with environmental and genetic factors. Dysbiosis of commensal bacteria and breakdown of the intestinal barrier integrity are considered to be major factors in the development of IBD. However, recent studies have indicated that genetic factors, including miRNA dysregulation, play a major role in the pathophysiology of IBD. Numerous miRNAs participate in the complex regulatory system of intestinal inflammation. Further, the number of molecular interactions seems to be uncountable; however, recent findings suggest the targeting of certain miRNAs as clinical biomarkers or treatment options. Additional *in vivo* studies should be conducted to validate data from *in vitro* studies and assess the practicality of manipulating miRNA expression in IBD.

## Figures and Tables

**Figure 1:** Biosynthesis of miRNA and the mechanism of action. miRNA: microRNA; RISC: RNA-induced silencing complex.

**Figure 2:** Intracellular interactions in intestinal homeostasis and inflammation. In intestinal homeostasis, commensal bacteria and dietary metabolites, such as RA and AhR ligands, induce immune tolerance through the action of Treg cells and anti-inflammatory cytokines, including IL-10 and TGF-β1. Various immune cells are recruited into the intestinal lamina propria but are not activated. However, IgA produced by plasma cells, and anti-microbial peptides, including REG3 and defensin, which are secreted from ILC3 and Th17 cells, prevent the pathogenic colonization of intestinal bacteria and invasion through the intestinal epithelium. In intestinal inflammation, direct invasion of commensal or pathogenic bacteria through the broken intestinal barrier causes inflammatory responses. Various immune cells and cytokines induce inflammatory reactions and augment anti-microbial activity. AhR: aryl hydrocarbon receptor; IFN: interferon; IL-: interleukin; ILC: innate lymphoid cell; NK T cell: natural killer T cell; PMN: polymorphonuclear leukocyte; RA: retinoic acid; REG3: Regenerating islet-derived protein 3; TGF β1: transforming growth factor β1; Th1: T helper type 1; Th2: T helper type 2; Th17: T helper type 17; TNF-α: tumor necrosis factor-α; Treg cell: regulatory T cell.

**Table 1:** Roles of miRNAs in the pathogenesis of inflammatory bowel disease

miRNAs	Targets	Functions	Ref.
**miRNAs that weaken the intestinal barrier**			
miR-21	PTEN/PI3K/Akt pathway	Increases the paracellular permeability of the intestinal epithelium	49
miR-122a	EGFR	Enhances the expression of zonulin and increases epithelial permeability	48
miR-191a, -212	ZO-1	Reduce the expression of ZO-1	44, 45
miR-675	Cadherin E, ZO-1	Destabilizes the mRNA of cadherin E and ZO-1	46
miR-874	Aquaporin 3	Decreases the expression of aquaporin 3	47
**miRNAs that strengthen the intestinal barrier**			
miR-93	PTK6	Reduces the expression of PTK6, and its downregulation attenuates epithelial injury	51
miR-200b	c-Jun, MLCK	Decreases epithelial damage induced by TNF-α in the intestinal epithelium	50
**miRNAs that increase inflammation**			
miR-21	MIP2, TNF-α	Increases the level of MIP2 and TNF-α	52
miR-124	AhR	Suppresses AhR expression and increases pro-inflammatory cytokine production	53
**miRNAs that decrease inflammation**			
miR-10a	IL-12/23p40	Downregulates the expression of IL-12/23p40 and Th1/Th17 cell responses	56
miR-141	CXCL12β	Inhibits CXCL12β-mediated leukocyte migration	57
miR-320	NOD2	Decreases the expression of NOD2	55
**miRNAs that enhance autophagy**			
miR-346	Vitamin-D receptor, GSK3B	Downregulates the expression of GSK3B, which increases ATG16L1	62
miR-665	XBP1, ORMDL3	Represses XBP1 and ORMDL3 expression	63
**miRNAs that inhibit autophagy**			
miR-20a	ATG16L1, SQSTM1	Downregulates BECN1, ATG16L1, and SQSTM1	64
miR-30C	ATG5, ATG16L1	Reduces the level of ATG5 and ATG16L1	65
miR-93, -106B	ATG16L1, PTEN	Suppress ATG16L1 expression and PTEN activity	66, 67
miR-122	NOD2, NF-κB	Inhibits NOD2 activity and increases NF-κB	69
miR-130a	p-mTOR	Increases the level of p-mTOR	71
miR-132, -223	FOXO3a	Downregulate FOXO3a, which enhances NF-κB signaling	72
miR-142-3p	ATG16L1	Decreases ATG16L1 mRNA and protein levels	68
miR-146b	SIAH2, FOXO3	Decreases SIAH2 and FOXO3 expression and activates the NF-κB pathway	74
miR-155	SHIP-1, FOXO3a	Increases Akt activity by decreasing SHIP-1, downregulates FOXO3a and enhances the NF-κB pathway	75, 76
miR-192	NOD2, NF-κB	Downregulates NOD2 expression and inhibits NF-κB activity	70
miR-196	LC3-II	Inhibits the accumulation of LC3-II	77
miR-320	NOD2	Reduces NOD2 expression	55

**Table 2:** miRNA signatures in inflammatory bowel disease

Sample type	Expression	miRNAs	Ref.
**Ulcerative colitis vs. healthy controls**			
Mucosal tissue	Upregulated	miR-7, miR-16, miR-20b, miR-21, miR-23a, miR-24, miR-26a, miR-26b, miR-29a, miR-29b, miR-31, miR-98, miR-99a, miR-126, miR-126*, miR-127-3p, miR-135b, miR-146a, miR-150, miR-155, miR-195, miR-203, miR-206, miR-324-3p, miR-424, miR-923, let-7a, let-7c, let-7d, let-7f, let-7g	80-86
	Downregulated	miR-141, miR-188-5p, miR-192, miR-215, miR-320a, miR-346, miR-375, miR-422b	80, 81, 87
Peripheral blood	Upregulated	miR-16, miR-19a, miR-21†, miR-28-5p, miR-101, miR-103-2, miR-142-5p, miR-151-5p, miR-155, miR-188-5p, miR-199a-5p, miR-223, miR-340, miR-362-3p, miR-375, miR-378, miR-422a, miR-494, miR-500, miR-501-5p, miR-532-3p, miR-769-5p, miR-874, miRplus-E1271	88, 98-100
	Downregulated	miR-21†, miR-31, miR-146a, miR-505	88, 99
**Crohn's disease vs. healthy controls**			
Mucosal tissues	Upregulated	miR-9, miR-21, miR-22, miR-26a, miR-29b, miR-29c, miR-30b, miR-31, miR-34c-5p, miR-101, miR-106a, miR-106b, miR-126*, miR-127-3p, miR-130a, miR-133b, miR-146a, miR-146b-5p, miR-150, miR-155, miR-181c, miR-196, miR-196a, miR-206, miR-324-3p, miR-375, miR-424	66, 77, 81, 85, 88
	Downregulated	miR-7, miR-375	88, 89
Peripheral blood	Upregulated	miR-16, miR-20a‡, miR-21‡, miR-23a, miR-29a, miR-30e‡, miR-93‡, miR-101, miR-106a, miR-107, miR-126, miR-140‡, miR-191, miR-192‡, miR-195‡, miR-199a-5p, miR-200c, miR-362-3p, miR-375, miR-484‡, miR-532-3p	88, 98, 101
	Downregulated	miR-21, miR-31, miR-146a, miR-155	88

*Complementary miRNA, †Upregulation from 98 and downregulation from 88, ‡From pediatric patients 101.

## Abbreviations

AhR: aryl hydrocarbon receptor
Akt: protein kinase B
ATG5: autophagy related 5
ATG16L1: autophagy related 16 like 1
BECN1: Beclin 1
CD: Crohn's disease
CD^+^: cluster of differentiation
CXCL: C-X-C motif chemokine ligand
DSS: Dextran sulfate sodium
EGFR: epidermal growth factor receptor
FOXO3 or FOXO3a: Forkhead box class O3
GM-CSF: granulocyte-macrophage colony-stimulating factor
GSK3B: glycogen synthase kinase 3 beta
GWAS: Genome-wide association studies
HDL: high-density lipoprotein
IBD: inflammatory bowel disease
IFN: interferon
Ig-: immunoglobulin
IL-: interleukin-
IL-12/23p40: p40 subunit of IL-12 and IL-23
ILC: innate lymphoid cell
LC3-II: the lipid modified form of microtubule-associated protein 1A/1B-light chain 3
MIP2: macrophage inflammatory protein 2
miRNA, miR: microRNA
MLCK: myosin light chain kinase
NF-κB: nuclear factor-light-chain-enhancer of activated B cells
NK T cell: natural killer T cell
NOD2: nucleotide-binding oligomerization domain-containing protein 2
ORMDL3: ORMDL sphingolipid biosynthesis regulator 3
p-Akt: phosphor-protein kinase B
PI3K: phosphoinositide 3-kinase
PIP2: phosphatidylinositol 4,5-biphosphate
PMN: polymorphonuclear leukocyte
p-mTOR: phosphorylated mammalian target of rapamycin
PTEN: phosphatase and tensin homolog
PTK6: protein tyrosine kinase 6
RA: retinoic acid
REG3: Regenerating islet-derived protein 3
RISC: RNA-induced silencing complex
RT-PCR: reverse-transcription polymerase chain reaction
SAA: serum amyloid A
SFB: segmented filamentous bacteria
SHIP-1: Src homology 2 domain containing inositol polyphosphate 5-phosphatase 1
SIAH2: Siah E3 ubiquitin protein ligase 2
SOCS3: suppressor of cytokine signaling 3
STAT: signal transducers and activators of transcription
SQSTM1: sequestosome 1
TAK1: transforming growth factor beta-activated kinase 1
TGF β1: transforming growth factor β1
Th1: T helper type 1
Th2: T helper type 2
Th17: T helper type 17
TNBS: 2,4,6-trinitrobenzen sulfonic acid
TNF-α: tumor necrosis factor-α
Treg cell: regulatory T cell
UC: ulcerative colitis
UTR: untranslated region
XBP1: X-box binding protein 1
ZO: zonula occludens

## References

[1] Guan Q (2019). A Comprehensive Review and Update on the Pathogenesis of Inflammatory Bowel Disease. J Immunol Res.

[2] Stidham RW, Higgins PDR (2018). Colorectal Cancer in Inflammatory Bowel Disease. Clin Colon Rectal Surg.

[3] Ng SC, Shi HY, Hamidi N, Underwood FE, Tang W, Benchimol EI (2018). Worldwide incidence and prevalence of inflammatory bowel disease in the 21st century: a systematic review of population-based studies. Lancet.

[4] Kaplan GG, Windsor JW (2021). The four epidemiological stages in the global evolution of inflammatory bowel disease. Nat Rev Gastroenterol Hepatol.

[5] Uniken Venema WT, Voskuil MD, Dijkstra G, Weersma RK, Festen EA (2017). The genetic background of inflammatory bowel disease: from correlation to causality. J Pathol.

[6] Ellinghaus D, Jostins L, Spain SL, Cortes A, Bethune J, Han B (2016). Analysis of five chronic inflammatory diseases identifies 27 new associations and highlights disease-specific patterns at shared loci. Nat Genet.

[7] de Lange KM, Moutsianas L, Lee JC, Lamb CA, Luo Y, Kennedy NA (2017). Genome-wide association study implicates immune activation of multiple integrin genes in inflammatory bowel disease. Nat Genet.

[8] Huang H, Fang M, Jostins L, Umićević Mirkov M, Boucher G, Anderson CA (2017). Fine-mapping inflammatory bowel disease loci to single-variant resolution. Nature.

[9] Liu JZ, van Sommeren S, Huang H, Ng SC, Alberts R, Takahashi A (2015). Association analyses identify 38 susceptibility loci for inflammatory bowel disease and highlight shared genetic risk across populations. Nat Genet.

[10] Park SC, Jeen YT (2019). Genetic Studies of Inflammatory Bowel Disease-Focusing on Asian Patients. Cells.

[11] Spehlmann ME, Begun AZ, Burghardt J, Lepage P, Raedler A, Schreiber S (2008). Epidemiology of inflammatory bowel disease in a German twin cohort: results of a nationwide study. Inflamm Bowel Dis.

[12] Halme L, Paavola-Sakki P, Turunen U, Lappalainen M, Farkkila M, Kontula K (2006). Family and twin studies in inflammatory bowel disease. World J Gastroenterol.

[13] Soroosh A, Koutsioumpa M, Pothoulakis C, Iliopoulos D (2018). Functional role and therapeutic targeting of microRNAs in inflammatory bowel disease. Am J Physiol Gastrointest Liver Physiol.

[14] O'Brien J, Hayder H, Zayed Y, Peng C (2018). Overview of MicroRNA Biogenesis, Mechanisms of Actions, and Circulation. Front Endocrinol (Lausanne).

[15] Lu Q, Wu R, Zhao M, Garcia-Gomez A, Ballestar E (2019). miRNAs as Therapeutic Targets in Inflammatory Disease. Trends Pharmacol Sci.

[16] Vidigal JA, Ventura A (2015). The biological functions of miRNAs: lessons from *in vivo* studies. Trends Cell Biol.

[17] Lozupone CA, Stombaugh JI, Gordon JI, Jansson JK, Knight R (2012). Diversity, stability and resilience of the human gut microbiota. Nature.

[18] Rooks MG, Garrett WS (2016). Gut microbiota, metabolites and host immunity. Nat Rev Immunol.

[19] Krause P, Morris V, Greenbaum JA, Park Y, Bjoerheden U, Mikulski Z (2015). IL-10-producing intestinal macrophages prevent excessive antibacterial innate immunity by limiting IL-23 synthesis. Nat Commun.

[20] Zigmond E, Bernshtein B, Friedlander G, Walker CR, Yona S, Kim KW (2014). Macrophage-restricted interleukin-10 receptor deficiency, but not IL-10 deficiency, causes severe spontaneous colitis. Immunity.

[21] Murdoch CC, Espenschied ST, Matty MA, Mueller O, Tobin DM, Rawls JF (2019). Intestinal Serum amyloid A suppresses systemic neutrophil activation and bactericidal activity in response to microbiota colonization. PLoS Pathog.

[22] Zhang G, Liu J, Wu L, Fan Y, Sun L, Qian F (2018). Elevated Expression of Serum Amyloid A 3 Protects Colon Epithelium Against Acute Injury Through TLR2-Dependent Induction of Neutrophil IL-22 Expression in a Mouse Model of Colitis. Front Immunol.

[23] Macpherson AJ, Yilmaz B, Limenitakis JP, Ganal-Vonarburg SC (2018). IgA Function in Relation to the Intestinal Microbiota. Annu Rev Immunol.

[24] Oliveira LM, Teixeira FME, Sato MN (2018). Impact of Retinoic Acid on Immune Cells and Inflammatory Diseases. Mediators Inflamm.

[25] Grizotte-Lake M, Zhong G, Duncan K, Kirkwood J, Iyer N, Smolenski I (2018). Commensals Suppress Intestinal Epithelial Cell Retinoic Acid Synthesis to Regulate Interleukin-22 Activity and Prevent Microbial Dysbiosis. Immunity.

[26] Pernomian L, Duarte-Silva M, de Barros Cardoso CR (2020). The Aryl Hydrocarbon Receptor (AHR) as a Potential Target for the Control of Intestinal Inflammation: Insights from an Immune and Bacteria Sensor Receptor. Clin Rev Allergy Immunol.

[27] Schanz O, Chijiiwa R, Cengiz SC, Majlesain Y, Weighardt H, Takeyama H (2020). Dietary AhR Ligands Regulate AhRR Expression in Intestinal Immune Cells and Intestinal Microbiota Composition. Int J Mol Sci.

[28] Yu LC (2018). Microbiota dysbiosis and barrier dysfunction in inflammatory bowel disease and colorectal cancers: exploring a common ground hypothesis. J Biomed Sci.

[29] Odenwald MA, Turner JR (2017). The intestinal epithelial barrier: a therapeutic target?. Nat Rev Gastroenterol Hepatol.

[30] Pickert G, Neufert C, Leppkes M, Zheng Y, Wittkopf N, Warntjen M (2009). STAT3 links IL-22 signaling in intestinal epithelial cells to mucosal wound healing. J Exp Med.

[31] Kotredes KP, Thomas B, Gamero AM (2017). The Protective Role of Type I Interferons in the Gastrointestinal Tract. Front Immunol.

[32] Shih VF, Cox J, Kljavin NM, Dengler HS, Reichelt M, Kumar P (2014). Homeostatic IL-23 receptor signaling limits Th17 response through IL-22-mediated containment of commensal microbiota. Proc Natl Acad Sci U S A.

[33] Coccia M, Harrison OJ, Schiering C, Asquith MJ, Becher B, Powrie F (2012). IL-1beta mediates chronic intestinal inflammation by promoting the accumulation of IL-17A secreting innate lymphoid cells and CD4(+) Th17 cells. J Exp Med.

[34] Zielinski CE, Mele F, Aschenbrenner D, Jarrossay D, Ronchi F, Gattorno M (2012). Pathogen-induced human TH17 cells produce IFN-gamma or IL-10 and are regulated by IL-1beta. Nature.

[35] Nowarski R, Jackson R, Gagliani N, de Zoete MR, Palm NW, Bailis W (2015). Epithelial IL-18 Equilibrium Controls Barrier Function in Colitis. Cell.

[36] Atreya R, Zimmer M, Bartsch B, Waldner MJ, Atreya I, Neumann H (2011). Antibodies against tumor necrosis factor (TNF) induce T-cell apoptosis in patients with inflammatory bowel diseases via TNF receptor 2 and intestinal CD14(+) macrophages. Gastroenterology.

[37] Pott J, Kabat AM, Maloy KJ (2018). Intestinal Epithelial Cell Autophagy Is Required to Protect against TNF-Induced Apoptosis during Chronic Colitis in Mice. Cell Host Microbe.

[38] Hunter CA, Jones SA (2015). IL-6 as a keystone cytokine in health and disease. Nat Immunol.

[39] Griseri T, McKenzie BS, Schiering C, Powrie F (2012). Dysregulated hematopoietic stem and progenitor cell activity promotes interleukin-23-driven chronic intestinal inflammation. Immunity.

[40] Griseri T, Arnold IC, Pearson C, Krausgruber T, Schiering C, Franchini F (2015). Granulocyte Macrophage Colony-Stimulating Factor-Activated Eosinophils Promote Interleukin-23 Driven Chronic Colitis. Immunity.

[41] Fan H, Wang A, Wang Y, Sun Y, Han J, Chen W (2019). Innate Lymphoid Cells: Regulators of Gut Barrier Function and Immune Homeostasis. J Immunol Res.

[42] Schaefer JS (2016). MicroRNAs: how many in inflammatory bowel disease?. Curr Opin Gastroenterol.

[43] Ma TY, Boivin MA, Ye D, Pedram A, Said HM (2005). Mechanism of TNF-{alpha} modulation of Caco-2 intestinal epithelial tight junction barrier: role of myosin light-chain kinase protein expression. Am J Physiol Gastrointest Liver Physiol.

[44] Wang L, Zhang R, Chen J, Wu Q, Kuang Z (2017). Baicalin Protects against TNF-alpha-Induced Injury by Down-Regulating miR-191a That Targets the Tight Junction Protein ZO-1 in IEC-6 Cells. Biol Pharm Bull.

[45] Tang Y, Zhang L, Forsyth CB, Shaikh M, Song S, Keshavarzian A (2015). The Role of miR-212 and iNOS in Alcohol-Induced Intestinal Barrier Dysfunction and Steatohepatitis. Alcohol Clin Exp Res.

[46] Zou T, Jaladanki SK, Liu L, Xiao L, Chung HK, Wang JY (2016). H19 Long Noncoding RNA Regulates Intestinal Epithelial Barrier Function via MicroRNA 675 by Interacting with RNA-Binding Protein HuR. Mol Cell Biol.

[47] Zhi X, Tao J, Li Z, Jiang B, Feng J, Yang L (2014). MiR-874 promotes intestinal barrier dysfunction through targeting AQP3 following intestinal ischemic injury. FEBS Lett.

[48] Zhang B, Tian Y, Jiang P, Jiang Y, Li C, Liu T (2017). MicroRNA-122a Regulates Zonulin by Targeting EGFR in Intestinal Epithelial Dysfunction. Cell Physiol Biochem.

[49] Zhang L, Shen J, Cheng J, Fan X (2015). MicroRNA-21 regulates intestinal epithelial tight junction permeability. Cell Biochem Funct.

[50] Shen Y, Zhou M, Yan J, Gong Z, Xiao Y, Zhang C (2017). miR-200b inhibits TNF-alpha-induced IL-8 secretion and tight junction disruption of intestinal epithelial cells *in vitro*. Am J Physiol Gastrointest Liver Physiol.

[51] Haines RJ, Beard RS Jr, Eitner RA, Chen L, Wu MH (2016). TNFalpha/IFNgamma Mediated Intestinal Epithelial Barrier Dysfunction Is Attenuated by MicroRNA-93 Downregulation of PTK6 in Mouse Colonic Epithelial Cells. PLoS One.

[52] Shi C, Liang Y, Yang J, Xia Y, Chen H, Han H (2013). MicroRNA-21 knockout improve the survival rate in DSS induced fatal colitis through protecting against inflammation and tissue injury. PLoS One.

[53] Zhao Y, Ma T, Chen W, Chen Y, Li M, Ren L (2016). MicroRNA-124 Promotes Intestinal Inflammation by Targeting Aryl Hydrocarbon Receptor in Crohn's Disease. J Crohns Colitis.

[54] Corridoni D, Arseneau KO, Cominelli F (2014). Functional defects in NOD2 signaling in experimental and human Crohn disease. Gut Microbes.

[55] Pierdomenico M, Cesi V, Cucchiara S, Vitali R, Prete E, Costanzo M (2016). NOD2 Is Regulated By Mir-320 in Physiological Conditions but this Control Is Altered in Inflamed Tissues of Patients with Inflammatory Bowel Disease. Inflamm Bowel Dis.

[56] Wu W, He C, Liu C, Cao AT, Xue X, Evans-Marin HL (2015). miR-10a inhibits dendritic cell activation and Th1/Th17 cell immune responses in IBD. Gut.

[57] Huang Z, Shi T, Zhou Q, Shi S, Zhao R, Shi H (2014). miR-141 Regulates colonic leukocytic trafficking by targeting CXCL12beta during murine colitis and human Crohn's disease. Gut.

[58] Yang Z, Klionsky DJ (2010). Eaten alive: a history of macroautophagy. Nat Cell Biol.

[59] Lapaquette P, Bringer MA, Darfeuille-Michaud A (2012). Defects in autophagy favour adherent-invasive Escherichia coli persistence within macrophages leading to increased pro-inflammatory response. Cell Microbiol.

[60] Wang S, Huang Y, Zhou C, Wu H, Zhao J, Wu L (2018). The Role of Autophagy and Related MicroRNAs in Inflammatory Bowel Disease. Gastroenterol Res Pract.

[61] Salem M, Ammitzboell M, Nys K, Seidelin JB, Nielsen OH (2015). ATG16L1: A multifunctional susceptibility factor in Crohn disease. Autophagy.

[62] Chen Y, Du J, Zhang Z, Liu T, Shi Y, Ge X (2014). MicroRNA-346 mediates tumor necrosis factor alpha-induced downregulation of gut epithelial vitamin D receptor in inflammatory bowel diseases. Inflamm Bowel Dis.

[63] Li M, Zhang S, Qiu Y, He Y, Chen B, Mao R (2017). Upregulation of miR-665 promotes apoptosis and colitis in inflammatory bowel disease by repressing the endoplasmic reticulum stress components XBP1 and ORMDL3. Cell Death Dis.

[64] Liu L, He J, Wei X, Wan G, Lao Y, Xu W (2017). MicroRNA-20a-mediated loss of autophagy contributes to breast tumorigenesis by promoting genomic damage and instability. Oncogene.

[65] Nguyen HT, Dalmasso G, Muller S, Carriere J, Seibold F, Darfeuille-Michaud A (2014). Crohn's disease-associated adherent invasive Escherichia coli modulate levels of microRNAs in intestinal epithelial cells to reduce autophagy. Gastroenterology.

[66] Lu C, Chen J, Xu HG, Zhou X, He Q, Li YL (2014). MIR106B and MIR93 prevent removal of bacteria from epithelial cells by disrupting ATG16L1-mediated autophagy. Gastroenterology.

[67] Li N, Miao Y, Shan Y, Liu B, Li Y, Zhao L (2017). MiR-106b and miR-93 regulate cell progression by suppression of PTEN via PI3K/Akt pathway in breast cancer. Cell Death Dis.

[68] Zhai Z, Wu F, Dong F, Chuang AY, Messer JS, Boone DL (2014). Human autophagy gene ATG16L1 is post-transcriptionally regulated by MIR142-3p. Autophagy.

[69] Chen Y, Wang C, Liu Y, Tang L, Zheng M, Xu C (2013). miR-122 targets NOD2 to decrease intestinal epithelial cell injury in Crohn's disease. Biochem Biophys Res Commun.

[70] Chuang AY, Chuang JC, Zhai Z, Wu F, Kwon JH (2014). NOD2 expression is regulated by microRNAs in colonic epithelial HCT116 cells. Inflamm Bowel Dis.

[71] Wang Y, Zhang X, Tang W, Lin Z, Xu L, Dong R (2017). miR-130a upregulates mTOR pathway by targeting TSC1 and is transactivated by NF-kappaB in high-grade serous ovarian carcinoma. Cell Death Differ.

[72] Kim HY, Kwon HY, Ha Thi HT, Lee HJ, Kim GI, Hahm KB (2016). MicroRNA-132 and microRNA-223 control positive feedback circuit by regulating FOXO3a in inflammatory bowel disease. J Gastroenterol Hepatol.

[73] Birnie KA, Yip YY, Ng DC, Kirschner MB, Reid G, Prele CM (2015). Loss of miR-223 and JNK Signaling Contribute to Elevated Stathmin in Malignant Pleural Mesothelioma. Mol Cancer Res.

[74] Nata T, Fujiya M, Ueno N, Moriichi K, Konishi H, Tanabe H (2013). MicroRNA-146b improves intestinal injury in mouse colitis by activating nuclear factor-kappaB and improving epithelial barrier function. J Gene Med.

[75] Rouquette-Jazdanian AK, Kortum RL, Li W, Merrill RK, Nguyen PH, Samelson LE (2015). miR-155 Controls Lymphoproliferation in LAT Mutant Mice by Restraining T-Cell Apoptosis via SHIP-1/mTOR and PAK1/FOXO3/BIM Pathways. PLoS One.

[76] Huang X, Shen Y, Liu M, Bi C, Jiang C, Iqbal J (2012). Quantitative proteomics reveals that miR-155 regulates the PI3K-AKT pathway in diffuse large B-cell lymphoma. Am J Pathol.

[77] Brest P, Lapaquette P, Souidi M, Lebrigand K, Cesaro A, Vouret-Craviari V (2011). A synonymous variant in IRGM alters a binding site for miR-196 and causes deregulation of IRGM-dependent xenophagy in Crohn's disease. Nat Genet.

[78] Melmed GY, Siegel CA, Spiegel BM, Allen JI, Cima R, Colombel JF (2013). Quality indicators for inflammatory bowel disease: development of process and outcome measures. Inflamm Bowel Dis.

[79] Canavese G, Villanacci V, Sapino A, Rocca R, Daperno M, Suriani R (2015). The diagnosis of inflammatory bowel disease is often unsupported in clinical practice. Dig Liver Dis.

[80] Wu F, Zikusoka M, Trindade A, Dassopoulos T, Harris ML, Bayless TM (2008). MicroRNAs are differentially expressed in ulcerative colitis and alter expression of macrophage inflammatory peptide-2 alpha. Gastroenterology.

[81] Fasseu M, Treton X, Guichard C, Pedruzzi E, Cazals-Hatem D, Richard C (2010). Identification of restricted subsets of mature microRNA abnormally expressed in inactive colonic mucosa of patients with inflammatory bowel disease. PLoS One.

[82] Takagi T, Naito Y, Mizushima K, Hirata I, Yagi N, Tomatsuri N (2010). Increased expression of microRNA in the inflamed colonic mucosa of patients with active ulcerative colitis. J Gastroenterol Hepatol.

[83] Feng X, Wang H, Ye S, Guan J, Tan W, Cheng S (2012). Up-regulation of microRNA-126 may contribute to pathogenesis of ulcerative colitis via regulating NF-kappaB inhibitor IkappaBalpha. PLoS One.

[84] Bian Z, Li L, Cui J, Zhang H, Liu Y, Zhang CY (2011). Role of miR-150-targeting c-Myb in colonic epithelial disruption during dextran sulphate sodium-induced murine experimental colitis and human ulcerative colitis. J Pathol.

[85] Lin J, Welker NC, Zhao Z, Li Y, Zhang J, Reuss SA (2014). Novel specific microRNA biomarkers in idiopathic inflammatory bowel disease unrelated to disease activity. Mod Pathol.

[86] Coskun M, Bjerrum JT, Seidelin JB, Troelsen JT, Olsen J, Nielsen OH (2013). miR-20b, miR-98, miR-125b-1*, and let-7e* as new potential diagnostic biomarkers in ulcerative colitis. World J Gastroenterol.

[87] Cai M, Chen S, Hu W (2017). MicroRNA-141 Is Involved in Ulcerative Colitis Pathogenesis via Aiming at CXCL5. J Interferon Cytokine Res.

[88] Schaefer JS, Attumi T, Opekun AR, Abraham B, Hou J, Shelby H (2015). MicroRNA signatures differentiate Crohn's disease from ulcerative colitis. BMC Immunol.

[89] Nguyen HT, Dalmasso G, Yan Y, Laroui H, Dahan S, Mayer L (2010). MicroRNA-7 modulates CD98 expression during intestinal epithelial cell differentiation. J Biol Chem.

[90] Ando Y, Mazzurana L, Forkel M, Okazaki K, Aoi M, Schmidt PT (2016). Downregulation of MicroRNA-21 in Colonic CD3+ T Cells in UC Remission. Inflamm Bowel Dis.

[91] Yang Y, Ma Y, Shi C, Chen H, Zhang H, Chen N (2013). Overexpression of miR-21 in patients with ulcerative colitis impairs intestinal epithelial barrier function through targeting the Rho GTPase RhoB. Biochem Biophys Res Commun.

[92] Thorlacius-Ussing G, Schnack Nielsen B, Andersen V, Holmstrom K, Pedersen AE (2017). Expression and Localization of miR-21 and miR-126 in Mucosal Tissue from Patients with Inflammatory Bowel Disease. Inflamm Bowel Dis.

[93] Wu F, Zhang S, Dassopoulos T, Harris ML, Bayless TM, Meltzer SJ (2010). Identification of microRNAs associated with ileal and colonic Crohn's disease. Inflamm Bowel Dis.

[94] Shi T, Xie Y, Fu Y, Zhou Q, Ma Z, Ma J (2017). The signaling axis of microRNA-31/interleukin-25 regulates Th1/Th17-mediated inflammation response in colitis. Mucosal Immunol.

[95] Zhang C, Zhao Z, Osman H, Watson R, Nalbantoglu I, Lin J (2014). Differential expression of miR-31 between inflammatory bowel disease and microscopic colitis. Microrna.

[96] Zahm AM, Hand NJ, Tsoucas DM, Le Guen CL, Baldassano RN, Friedman JR (2014). Rectal microRNAs are perturbed in pediatric inflammatory bowel disease of the colon. J Crohns Colitis.

[97] Guo Z, Wu R, Gong J, Zhu W, Li Y, Wang Z (2015). Altered microRNA expression in inflamed and non-inflamed terminal ileal mucosa of adult patients with active Crohn's disease. J Gastroenterol Hepatol.

[98] Paraskevi A, Theodoropoulos G, Papaconstantinou I, Mantzaris G, Nikiteas N, Gazouli M (2012). Circulating MicroRNA in inflammatory bowel disease. J Crohns Colitis.

[99] Wu F, Guo NJ, Tian H, Marohn M, Gearhart S, Bayless TM (2011). Peripheral blood microRNAs distinguish active ulcerative colitis and Crohn's disease. Inflamm Bowel Dis.

[100] Duttagupta R, DiRienzo S, Jiang R, Bowers J, Gollub J, Kao J (2012). Genome-wide maps of circulating miRNA biomarkers for ulcerative colitis. PLoS One.

[101] Zahm AM, Thayu M, Hand NJ, Horner A, Leonard MB, Friedman JR (2011). Circulating microRNA is a biomarker of pediatric Crohn disease. J Pediatr Gastroenterol Nutr.

[102] Viennois E, Zhao Y, Han MK, Xiao B, Zhang M, Prasad M (2017). Serum miRNA signature diagnoses and discriminates murine colitis subtypes and predicts ulcerative colitis in humans. Sci Rep.

[103] Jensen MD, Andersen RF, Christensen H, Nathan T, Kjeldsen J, Madsen JS (2015). Circulating microRNAs as biomarkers of adult Crohn's disease. Eur J Gastroenterol Hepatol.

[104] Gallo A, Tandon M, Alevizos I, Illei GG (2012). The majority of microRNAs detectable in serum and saliva is concentrated in exosomes. PLoS One.

[105] Vickers KC, Palmisano BT, Shoucri BM, Shamburek RD, Remaley AT (2011). MicroRNAs are transported in plasma and delivered to recipient cells by high-density lipoproteins. Nat Cell Biol.

[106] Chen WX, Ren LH, Shi RH (2014). Implication of miRNAs for inflammatory bowel disease treatment: Systematic review. World J Gastrointest Pathophysiol.

[107] Tian Y, Xu J, Li Y, Zhao R, Du S, Lv C (2019). MicroRNA-31 Reduces Inflammatory Signaling and Promotes Regeneration in Colon Epithelium, and Delivery of Mimics in Microspheres Reduces Colitis in Mice. Gastroenterology.

[108] Neudecker V, Haneklaus M, Jensen O, Khailova L, Masterson JC, Tye H (2017). Myeloid-derived miR-223 regulates intestinal inflammation via repression of the NLRP3 inflammasome. J Exp Med.

[109] Cheng X, Zhang X, Su J, Zhang Y, Zhou W, Zhou J (2015). miR-19b downregulates intestinal SOCS3 to reduce intestinal inflammation in Crohn's disease. Sci Rep.

[110] Yang J, Zhou CZ, Zhu R, Fan H, Liu XX, Duan XY (2017). miR-200b-containing microvesicles attenuate experimental colitis associated intestinal fibrosis by inhibiting epithelial-mesenchymal transition. J Gastroenterol Hepatol.

[111] Zhang M, Viennois E, Prasad M, Zhang Y, Wang L, Zhang Z (2016). Edible ginger-derived nanoparticles: A novel therapeutic approach for the prevention and treatment of inflammatory bowel disease and colitis-associated cancer. Biomaterials.

[112] Fukata T, Mizushima T, Nishimura J, Okuzaki D, Wu X, Hirose H (2018). The Supercarbonate Apatite-MicroRNA Complex Inhibits Dextran Sodium Sulfate-Induced Colitis. Mol Ther Nucleic Acids.

